# Early Warning of Basketball Injury Risk Based on Attribute Reduction Algorithm

**DOI:** 10.1155/2022/6981246

**Published:** 2022-04-13

**Authors:** Peng Wang, Seungsoo Baek

**Affiliations:** Department of Sport & Health Care, College of Culture and Arts, Sangmyung University, Seoul 03016, Republic of Korea

## Abstract

Basketball is one of the students' favorite ball games, and it is also one of the most popular sports for college students to carry out after class. Especially in recent years, with the spread of NBA culture around the world and the extensive development of CUBA in domestic colleges and universities, Yao Ming has appeared in China to compete in the NBA and achieve brilliant achievements. With the increasing investment in the number of basketball venues, basketball itself, as a sport with low dependence on venues, equipment, and people, has the characteristics of economy, convenience, and remarkable sports effect compared with other sports. College students' basketball skills, basketball awareness, and love for basketball are increasing day by day. Attribute reduction algorithm is one of the core contents of knowledge discovery, which describes whether every attribute in the attribute set of information system is necessary and how to delete unnecessary knowledge. Based on the attribute reduction algorithm, this paper studies the early warning of basketball injury risk. The basketball injury can not only make athletes unable to participate in training or competition, but even cripple or lose their lives, which hinders the normal development of sports. Therefore, we should make a comprehensive and objective analysis of sports training to find out the causes of sports injuries, so as to prevent sports injuries. This algorithm takes the attribute frequency as the heuristic information and solves the attribute selection problem when the attribute frequency is the same.

## 1. Introduction

Basketball is one of the sports with high popularity and is loved by college students in college students' sports activities. It plays a positive role in improving students' physiological function, enhancing students' physique, exercising students' good mood and will quality, and cultivating students' good social interpersonal relationship. Basketball is one of the students' favorite ball games and one of the most popular extracurricular sports for college students. Especially in recent years, NBA culture has spread all over the world, CUBA has been widely carried out in domestic colleges and universities, Yao Ming has entered the NBA and made brilliant achievements in China, and college students' basketball technology, basketball consciousness, and love for basketball are increasing day by day [1]. With the increasing investment in the number of basketball venues, basketball itself, as a sport with low dependence on venues, equipment, and people, has the characteristics of economy, convenience, and remarkable sports effect compared with other sports. It attracts the participation of basketball lovers [2, 3]. However, basketball is also a kind of sports with high intensity and fierce confrontation. Because college students do not have a clear understanding of injury risk factors in basketball, they do not pay enough attention to the prevention of sports injury or lack the concept of prevention, resulting in sports injury in basketball, which has a lot of adverse effects on college students' campus life [4]. During the development of sports events, injury and illness is an important factor affecting athletes' performance, which directly determines whether they can give full play to their own strength. However, the sports injury in college basketball is also increasing, which affects their learning, training, and life. Therefore, it is very important to study the time period, location, type, and cause of sports injury of basketball lovers and actively take preventive measures.

In view of this, based on the attribute reduction algorithm, this paper studies the screening methods of indicators causing athletes' injuries, and then, after the screening is completed, it can realize the effective early warning of athletes' injuries and reduce the probability of athletes' injuries [5, 6]. Through the above research, it can provide the basis and reference for the current scientific prediction and evaluation of athletes' injuries [7]. Rough set theory was put forward by Polish mathematician Z. Pawlak in 1982. As one of the core contents of knowledge discovery in attribute reduction algorithm, it describes whether every attribute in the attribute set of information system is necessary and how to delete unnecessary knowledge [8, 9]. Attribute reduction algorithm theory is a new mathematical theory to deal with inaccurate, incomplete, and incompatible knowledge, which has been widely used in artificial intelligence, pattern recognition, data mining, and intelligent decision-making and other fields [10, 11]. In the theory of attribute reduction algorithm, attribute reduction is one of the important research contents. At present, the attribute reduction algorithms are mainly based on information entropy, discernibility matrix, discernibility matrix, and so on, each of which has achieved considerable results in some problems. Many scholars have put forward reduction algorithms using kernel and attribute importance, which use kernel as the starting point of reduction calculation and attribute importance as the heuristic rule to calculate the minimum reduction.

The main advantage of attribute reduction algorithm in basketball injury risk early warning is that it does not need the support of experience and additional data but only needs to mine the potential relationship and rules of the problem based on the classification of data [12, 13]. This algorithm takes the attribute frequency as the heuristic information and solves the attribute selection problem when the attribute frequency is the same. That is, the judgment standard of attribute importance with the same attribute frequency is proposed. It solves the problem that the importance degree is the same when the attribute frequency is used as the attribute importance measure in the discernibility matrix [14, 15].

## 2. Related Work

### 2.1. Research Status at Home and Abroad

Bittencourt et al. [16] put forward that, in view of the antagonism and fierce competition of basketball, college students' basketball injury risk factors can be divided into two types, namely, controllable risk factors and uncontrollable risk factors. Cibin et al. [17] studied the risk factors and characteristics of college students' sports injuries in basketball by big data analysis method and provided theoretical guidance and suggestions for college students in basketball, so that college students could avoid and reduce injuries as much as possible, improve their physical quality, and provide guarantee for the smooth development of college students' basketball. Räisänen et al. [18] research shows that, in this study, functional action screening (FMS) is used to assess the risk of football injury for male football players in colleges and universities. To observe the influence of 12-week practice on FMS score, biomechanical characteristics and dynamic balance ability of college male football players is monitored. The results show that exercise can significantly improve the functional defects related to sports injuries of male basketball players. Räisänen et al. [18] pointed out that, in basketball, adequate preparation plays a key role in preventing muscle and joint injuries. Doing adequate preparation before exercise, raising the temperature of muscles, and reducing the viscosity of muscles can reduce the possibility of muscle strain during exercise. Castro et al. [19] divided 30 FAI male college students into experimental group and control group by big data analysis method, with 15 students in each group. The experimental group received rehabilitation training, while the control group received elastic belt + balance pad rehabilitation training. After 16 weeks of experiment, it was concluded that the exercise could significantly improve the ankle muscle strength, proprioception, and dynamic balance ability of lower limbs of FAI students. Wang's [20] research shows that the excitement of the central nervous system of human body is a slow process, and the physiological inertia of internal organs also exists. In order to adapt to the relatively intense and intense basketball, it is necessary to carry out sufficient preparation activities to slowly mobilize the excitement of the nervous system and gradually overcome the physiological inertia of various internal organs. Liang et al. [21] pointed out that basketball requires participants' physical qualities, including strength, speed, endurance, coordination, and sensitivity, which are necessary to complete the difficult skills in basketball technology. However, some students' physical qualities are not very good, coupled with the lack of systematic training, but they want to try beautiful but difficult basketball skills, which often makes it difficult to complete the difficult basketball skills normally and greatly increase. Ma et al. [22], through the method of big data analysis, show that fatigue will cause the decline of various functions of the body, the fatigue of the nervous system will cause the change of neuromuscular control mechanism, and the sensory feedback of proprioceptors to joints and muscles will also decrease. At this time, the adjustment ability of the nervous system to fine basketball movements will also decrease, which will easily lead to the change of basketball technical movements and cause sports injuries. Wei et al. [23] research shows that 42 college male basketball players are randomly divided into control group (*n* = 21) and intervention group (*n* = 21). The intervention group adopts exercise and the control group adopts routine warm-up exercise. After the experiment twice a week for 12 weeks, the research conclusion shows that 12 weeks of practice can significantly improve the power characteristics and dynamic balance ability of men's basketball players, reduce the functional defects related to sports injury, and have a significant effect on reducing the injury risk of men's basketball players. According to Gao et al. [24], students' love of basketball can be promoted to master correct basketball skills by strengthening the training and guidance of basic skills, form the correct technical “dynamic shaping” to make it conform to the physiological and anatomical characteristics of the human body and the mechanical principle of sports, so as to improve the students' physical quality and the ability of confrontation and competition, and prevent sports injuries caused by technical action errors.

### 2.2. Research Status of Basketball Injury Prevention Based on Attribute Reduction Algorithm

Based on attribute reduction algorithm, this paper studies the early warning of basketball sports injury risk. Many college students do not understand or ignore the role of preparation activities because of lack of sports healthcare knowledge, and they do not do enough preparation activities. Some of them simply do not do preparation activities, and they engage in intense basketball activities without fully mobilizing their various functions, which increases the possibility of sports injury. In the research of basketball injury prevention, some scholars have begun to apply some training methods to warm-up activities to verify their effectiveness in preventing basketball injury. And the prevention plan can effectively reduce the incidence of sports injuries. However, the research on sports injury prevention in China mainly finds out the situation and causes of basketball sports injuries through questionnaires, documents, and other methods and puts forward preventive measures, including strengthening self-prevention awareness, improving technical level, and strengthening the management of sports venues and facilities, but does not put forward concrete and substantive exercise methods to prevent sports injuries. This paper explores the effect of injury risk intervention for young basketball players, puts forward new directions and ideas for the development of basketball injury prevention practice methods, achieves the purpose of reducing youth basketball injury, enriching basketball injury prevention methods, and enriching basketball warm-up methods, and provides valuable reference basis and direction for basketball injury prevention in the future.

## 3. Principle and Model of Attribute Reduction Algorithm

Reduction is one of the important concepts of rough sugar set for data analysis. At present, there are not only a large number of records, but also many fields such as characteristics and variables in various database storage, which leads to high data complexity. The reduction of information system fields in rough set is attribute reduction, while a large number of records are regarded as value reduction. At present, the attribute reduction algorithm of rough set theory has been gradually applied in sports competition, mainly through mining a large number of athletes' competition and training data, so as to analyze and predict athletes' status and training effect and thus provide data support for scientifically and reasonably making training or competition plans. With the increasing amount of data, attribute reduction ratio reduction is more effective. If we want to improve people's understanding of all kinds of knowledge in information system, we must reduce a lot of redundancy and simplify the complexity of database structure before knowledge acquisition. At present, in the field of sports competition, common attribute reduction algorithms include attribute reduction algorithm based on discernibility matrix, attribute reduction algorithm based on dependency, attribute reduction algorithm based on mutual information, and so on. Attribute reduction based on attribute importance is a reduction algorithm proposed to reduce the complexity of reduction results. Based on the general attribute reduction algorithm, that is, the attribute reduction algorithm based on positive domain, it calculates the core attributes of conditional attributes for decision attributes. Then, an attribute importance method is proposed by using the attribute dependence in the rough sugar set. In the process of reduction, the attributes with high importance except the core attributes in the information system are added to the reduction set in turn until the whole information system is traversed. The algorithm flowchart is shown in Figure 1.

The idea of the reduction algorithm based on attribute importance is simple. Taking the attribute core as the starting point of reduction, the attributes with high attribute importance are added to the reduction set until the termination conditions are met. The calculation amount of this algorithm is relatively small and the time complexity is relatively low. However, the algorithm can only get a reduction of the information system and can not guarantee that the reduction is the smallest. General reduction algorithm is also called attribute reduction based on positive field. It is the most intuitive algorithm in attribute reduction algorithm; that is, delete an attribute from the decision table and then compare the equivalence relationship between the existing decision table and the original decision table. If it is the same as the original decision table, it is considered that the deleted attribute is an unnecessary attribute and so on. The occurrence of sports injury is not caused by a simple reason but often the result of the joint action of multiple factors. In order to make a more accurate early warning of sports injury, we must first clarify what factors will directly or indirectly lead to sports injury. The risk factors inducing sports injury are generally divided into internal factors and external factors. These factors can also be divided into controllable factors and uncontrollable factors. The internal risk factors are often uncontrollable. The dynamic chain model of sports injury etiology is shown in Figure 2.

In the early warning of athletes' injuries and injuries, it is necessary to construct emergency decisions and adopt different methods according to different injuries. Because of the different attributes of the data causing athletes' injuries, the range dimensions of the data are also different, so the interval values between the range values are correspondingly different. Build a mathematical model of quantitative attributes.

The dimensionless value *v*′*c* of the attribute *c*_*j*_ can be expressed as

(1) $$\begin{array}{c} \upsilon_{j}^{\prime }=\left\{\begin{array}{cc} 0, & \upsilon_{j}\leq \upsilon_{\min j},\\ \frac{\upsilon_{j}-\upsilon_{\min j}}{\upsilon_{\max j}-\upsilon_{\min j}}, & \upsilon_{\min j}<\upsilon_{j}<\upsilon_{\max j},\\ 1, & \upsilon_{j}\leq \upsilon_{\min j}, \end{array}\right) \end{array}$$

(2) $$\begin{array}{c} \upsilon_{j}^{\prime }=\left\{\begin{array}{cc} 1, & \upsilon_{j}\leq \upsilon_{\max j},\\ \frac{\upsilon_{\max}-\upsilon_{j}}{\upsilon_{\max j}-\upsilon_{\min j}}, & \upsilon_{\min j}<\upsilon_{j}<\upsilon_{\max j},\\ 0, & \upsilon_{j}\geq \upsilon_{\max j}. \end{array}\right) \end{array}$$

Formulas (1) and (2) represent application models in different situations. This depends on the different attributes. For example, when athletes are in competitive events, formula (1) can be applied. In normal training, formula (2) can be applied.

The evaluation index set is expressed by *A*, where *A* = (good, better, fair, poor, poor).

Suppose again:

*R*_*j*_ is expressed as membership vector, and data set is expressed as

(3) $$\begin{array}{c} r_{j}=\left(r_{j1},r_{j2},r_{j3},r_{j4},r_{j5}\right), \end{array}$$

where RJ represents the membership vector corresponding to the index evaluation set a. *R*_*e*_ hypothesis

(4) $$\begin{array}{c} B={\left(B_{1},B_{2},B_{3},B_{4},B_{5}\right)}^{T}. \end{array}$$

*B*_*i*_ is used as the scale element corresponding to the *i*-level evaluation in data set *B*. Through data set *B*, the data membership vector representing athlete injury can be effectively synthesized into scalar, expressed as

(5) $$\begin{array}{c} V=r_{j}\times B, \end{array}$$

where *V* is the quantitative value of qualitative evaluation index of athlete injury data under the given scale *B*.

According to the different membership degrees, the Hamming distance of two different fuzzy data set values can be defined, respectively. When the distance is not greater than the threshold of rating the degree of athlete's injury, it is expressed as having a certain correlation with causing athlete's injury, and the correlation value is expressed by *R*.

The similarity calculation formula is shown in the following formula:

(6) $$\begin{array}{c} x_{a}Rx_{b}=\left(x_{\alpha },x_{b}\right)\in U*U\left|\frac{1}{m}\sum_{j=1}^{m}\left|\upsilon_{aj}^{\prime }-\upsilon_{bj}^{\prime }\right|\leq \alpha \right|, \end{array}$$

where *x*_*i*_ ∈ *U*(*i*=1,2,…, *n*); ∀*x*_*α*_, *x*_*b*_, ∀*c*_*j*_∈ athlete's strain data attribute *C*, *j*=1,2,…, *m* is expressed as the attribute value of the object *x*_*i*_ in the data set in the data attribute *c*_*j*_; *υ*_*ij*_′ represents the quantified value of athletes' injuries. Through the above formula, 1 − *α* is expressed as the similarity between athlete strain data *x*_*α*_ and athlete strain data *x*_*b*_. *R* is used to express the fuzzy similarity relationship between reflexivity and symmetry of athletes' strain data, and then it is expressed by formula as follows:

(7) $$\begin{array}{c} R\left(x_{i}\right)=\left\{x_{\alpha }\in U\left|\frac{1}{m}\sum_{j=1}^{m}\left|\upsilon_{\alpha j}^{\prime }-\upsilon_{bj}^{\prime }\right|\leq \alpha \right|,\;j=1,2,\ldots ,m\right\}, \end{array}$$

where *x*_*i*_ represent that data elements constitute the athlete's strain; *R*(*x*_*i*_) is expressed as a fuzzy similarity formula with *x*_*i*_.

(8) $$\begin{array}{c} R={\left(r_{ij}\right)}_{n\times m}. \end{array}$$

Suppose that the ideal evaluation scheme for athletes' injuries is as follows:

(9) $$\begin{array}{c} G=\left(g_{1},g_{2},\ldots ,g_{m}\right). \end{array}$$

In formula (9)

(10) $$\begin{array}{c} g_{j}=\overset{\max r_{ij}}{1\leq i\leq n}. \end{array}$$

Dis(*x*_*i*_, *G*) is expressed as the closeness degree, which is expressed as the weighted Hamming distance between *x*_*i*_ and *g*. When estimating athletes' injuries and injuries, the probability of each type of reduction sets is almost the same. The total closeness indicates the weighted sum of closeness of different technical schemes in the reduction sets. The calculated value of the weighted sum is inversely proportional to the superiority of the schemes. Specifically, the smaller the calculated value of the weighted sum, the better the superiority of the schemes.

In the theoretical model, external factors are defined as “initiating factors.” When it appears, athletes with injury tendency with internal injury factors will be called “injury prone people,” and they will be more prone to injury. However, only the appearance and interaction of internal and external factors alone are not enough to induce athletes to have injuries but to make them become “susceptible people.” Under certain conditions, they will have sports injuries. In this paper, the attribute reduction algorithm is applied to the athlete training information system, which can effectively obtain the internal or external parameters of athletes in sports. These parameters are analyzed through the injury early warning model to prevent the occurrence of athletes' injuries to the greatest extent. The system includes four layers: data layer, feature layer, attribute reduction algorithm layer, and decision layer. The evaluation of athletes' muscle strain degree is based on the information acquisition and processing of athletes' human movement process. Therefore, the main research of this paper is how to use attribute reduction algorithm to evaluate athletes' muscle strain. The overall system architecture design is shown in Figure 3.

In the data layer, it mainly realizes the collection of athletes' parameter information. The information collected is diverse, including internal factors and external factors. Internal factors include athletes' mood, physical condition, physique, improvisation, sports skills, and other parameters. External factors include parameters such as competition venue, on-the-spot accidents, weather, environment, competition order, competition rules, equipment, and so on. The reduction algorithm based on discernibility matrix is to filter out the attributes with only unique elements by constructing discernibility matrix, take this attribute as the core, judge other sets containing several attribute items, and then further construct the discernibility function on this basis, and make disjunction and conjunction.

## 4. Basketball Injury Risk Early Warning

### 4.1. Prevention of Basketball Injury Risk Factors Based on Attribute Reduction Algorithm

Strengthen college students' learning of basketball healthcare knowledge, make college students fully realize the role of preparatory activities in the prevention of sports injury by attribute reduction algorithm, and cultivate college students' good habit of preparatory activities before basketball. At present, in the field of sports competition in China, after collecting the relevant data of injury and early warning of basketball players, we mainly use the methods of questionnaire, referring to expert experience and consulting relevant literature to analyze the data, so as to determine the potential factors causing injury and injury of athletes and evaluate the early warning level of these factors, as a basis for further determining the potential relationship between these factors and early warning level. Focus on the parts with injury history, vulnerable parts, and parts with large local load. At the same time, based on attribute reduction algorithm, in order to recover fatigue quickly, we should carry out effective relaxation activities in time after exercise and strengthen nutrition and rest at the same time, so as to quickly recover the body state and avoid the accumulation of exercise fatigue. In this regard, in order to find different injury investigation indicators of athletes, taking track and field athletes in a city as a case, the injury early warning indicators for track and field athletes are determined by consulting data and literature and referring to expert experience. For this, this paper selects 21 indicators, including age, physical fitness index, and subjective emotion. See Table 1 for details.

In the above indicators, all factors that may affect athletes' injuries and injuries are involved, so as to summarize them comprehensively. Through the above selection, it lays a foundation for the subsequent judgment of athletes' injuries and injuries. In this paper, 10 basketball players in a city were randomly selected as test source data, and then the simulation test results were compared with the actual values to verify the feasibility of the method proposed in this paper. The final output of the simulation test is shown in Table 2.

From the simulation test results shown in the table, it can be seen that the prediction results with small error with the actual value can be obtained through the method proposed in this paper, which meets the accuracy requirements of basketball players' injury early warning in the field of sports competition. It also shows that the test results are more accurate in terms of accuracy. It can be concluded that, in the evaluation of athletes' injuries, the main judgment indicators are the intensity of training, the degree of injury recovery, psychological state, and so on. These indicators are consistent with the interview records of athletes' injuries, which shows that the indicators obtained by the attribute reduction algorithm are consistent with the reality, feasible, and accurate. As basketball has certain requirements for all aspects of college students' physical quality, we should comprehensively develop college students' physical quality to meet the requirements of basketball in terms of speed, strength, endurance, and flexibility and strengthen the practice of muscle strength and joint flexibility in vulnerable parts, to avoid sports injury caused by poor physical fitness.

### 4.2. Experimental Results and Analysis

Strengthen safety education and enhance the awareness of the significance of injury prevention. Teachers should fully understand the importance of injury prevention and take necessary measures to strengthen safety education. Teachers are not only the organizers of teaching, but also the transmitters of sports knowledge, technology, and skills. If teachers themselves lack knowledge of injuries, do not pay attention to students' safety, and take an irresponsible attitude, they will not only fail to complete the teaching tasks well, but also be prone to injuries. The key to prevent sports injuries lies in PE teachers. Therefore, it is necessary to improve PE teachers' awareness of safety precautions, make full use of various forms to enable students to master reasonable methods of preparation activities, guide students to do full preparation activities, and cultivate students' good habit of doing preparation activities before sports. In the experiment, the test within a certain time range was selected, assuming that the test was carried out within 95 s, and three experiments were carried out for comparison, through machine learning algorithm, decision tree algorithm, genetic algorithm, and this algorithm. During the test, a wounded person was selected to have poor performance due to the weather. The experimental results are shown in Figures 4–6.

Through the comparison of the above algorithms, for different basketball player injury data sets, a number of reduction condition attributes of the above four different algorithms are used. Under the same circumstances and at the same time, the error data are different. The algorithm error data in this study is the smallest and the error data is small, which indicates that the sensitivity of early warning is high. In the process of basketball competition, it needs strong outbreak and speed. In order to deal with emergencies on the basketball court and give timely and effective response, we need high sensitivity and so on. At the same time, poor flexibility is often prone to muscle and ligament strain during exercise. As college students come from different regions, their physical quality will also be uneven, some even poor, which will cause damage in the relatively fierce confrontational basketball game. The purpose of preparatory activities is to improve the excitability of the central nervous system and overcome the inertia of human function through a variety of exercises. Teachers should choose some targeted preparation activities according to the characteristics that basketball is easy to cause injury and let students understand the significance of doing preparation activities.

Next, we will compare and analyze the sensitivity of early warning after adopting this research scheme. Assuming that the abnormality is set in 10 aspects such as joint flexibility, joint protection measures, mental state, joint stability, and training load, machine learning algorithm, decision tree algorithm, genetic algorithm, and the algorithm in this paper are used for two comparative analysis, respectively, to observe the curve of sensitivity change at any time, as shown in Figures 7 and 8.

As shown in Figures 7 and 8, the speed of the calculation model is mainly based on the test data within a certain period of time; that is, the sensitivity and reaction speed of the calculation model change with time. The longer the running time, the faster the reaction of the calculation model and the better the calculation speed, and correspondingly, the higher the sensitivity. During the whole experiment, the method studied in this paper has higher calculation speed and higher sensitivity than the other two methods in the same time. The attribute reduction algorithm based on mutual information mainly describes the definition and calculation of rough set based on information theory. Specifically, it starts with the conditional attribute as the core attribute in the decision table, filters the attribute set, and adds the most important content into the core attribute until the mutual information is equal.

## 5. Conclusions

Basketball players will suffer from injuries due to many factors in training and competition. Aiming at this problem, this paper proposes a combination of attribute reduction algorithm and basketball injury risk early warning method. This method can extract the key indicators of athletes' injury factors efficiently and accurately and evaluate their early warning level, so as to effectively obtain the injury situation of athletes and reduce the probability of basketball players' injuries again, which provides a reference for the current scientific and information analysis of athletes' injuries. In order to speed up the scientific basketball training, from the perspective of multidisciplinary, based on the systematic understanding of the characteristics of basketball training, this paper defines the influence of various elements causing basketball players' sports injury on sports injury and realizes a reasonable and effective reduction algorithm combined with the attribute reduction method in rough set theory. It is used to reduce the injury indicators affecting the injury of basketball players, mine the factors with high contribution rate to basketball injury, and apply it to the establishment of track and field injury early warning model, which provides a new method for the prevention of sports injury of basketball players. At the same time, based on attribute reduction algorithm, in order to recover fatigue quickly, we should carry out effective relaxation activities in time after exercise and strengthen nutrition and rest at the same time, so as to quickly recover the body state and avoid the accumulation of exercise fatigue. In major sports events, coaches can use the method of this study to quickly make judgments from complex sports events. Therefore, it is necessary to improve PE teachers' awareness of safety precautions, make full use of various forms to enable students to master reasonable methods of preparation activities, guide students to do full preparation activities, and cultivate students' good habit of doing preparation activities before sports.

## Figures and Tables

**Figure 1:** Flowchart of attribute importance reduction algorithm.

**Figure 2:** Dynamic chain model of sports injury etiology.

**Figure 3:** System overall.

**Figure 4:** Schematic diagram of error curve.

**Figure 5:** Schematic diagram of error curve.

**Figure 6:** Schematic diagram of error curve.

**Figure 7:** Schematic diagram of calculation percentage of reaction time.

**Figure 8:** Schematic diagram of calculation percentage of reaction time.

**Table 1:** Attribute reduction algorithm for early warning index of basketball players' injury.

Sign	Index	Sign	Index	Sign	Index
*A*	Age	*B*	Sports grade	*C*	Menstrual cycle
*D*	Physical fitness index	*E*	History of injuries	*F*	Degree of recovery from past injuries
*G*	Joint flexibility	*H*	Joint stability	*I*	Strength comparison of front and back thigh muscles
*J*	Comparison of left and right thigh circumference	*K*	Physical coordination	*L*	Arch shape of foot
*M*	Engineering level	*N*	Action standard degree	*O*	Joint protection
*P*	Intensity of training	*Q*	Training ground	*R*	Training plan
*S*	Equipment replacement	*T*	Physical fatigue	*U*	Subjective emotion

**Table 2:** Final output result of simulation test.

Test result	Actual value	Test result	Actual value	Test result	Actual value
1.0258	1	2.1245	2	3.1235	2
2.1354	1	1.1236	2	1.1236	2
2.1568	2	1.1354	1	1.0248	1
2.0034	2	2.9426	2	2.0745	3

## Data Availability

The datasets used and/or analyzed during the current study are available from the corresponding author on reasonable request.
